The article "Chrysophanol exerts a protective effect against sepsis-induced acute myocardial injury through modulating the microRNA-27b-3p/Peroxisomal proliferating-activated receptor gamma axis" was retracted in 2026. Reasons: concerns about the data; concerns about the results or conclusions.

# Chrysophanol exerts a protective effect against sepsis-induced acute myocardial injury through modulating the microRNA-27b-3p/Peroxisomal proliferating-activated receptor gamma axis

**DOI:** 10.1080/21655979.2022.2063560

**Published:** 2022-05-21

**Authors:** Haiyan Zhao, Yuping Wang, Xiaolin Zhu

**Affiliations:** a Dry Treatment Department of Critical Care Medicine, The First Affiliated Hospital of Kunming Medical University, Kunming, Xishan, China; b Department of Critical Care Medicine, The First Affiliated Hospital of Kunming Medical University, Kunming, Xichang, China; c Dry Treatment Intensive Care Unit, The First Affiliated Hospital of Kunming Medical University, Kunming, Xichang, China

**Keywords:** sepsis, myocardial injury, chrysophanol, inflammation, microRNA-27b-3p

## Abstract

Sepsis, a leading contributor to the death of inpatients, results in severe organ dysfunction as complications. The heart is one of the major organs attacked by sepsis, and the effective control of the inflammatory cascade reaction in sepsis is of great significance in alleviating sepsis-associated acute myocardial injury (S-AMI). Chrysophanol, a natural anthraquinone, has been discovered to carry anti-inflammatory effects. The aim of this paper is to probe the impact of Chrysophanol on S-AMI. An S-AMI model was engineered in rats via CLP. Pathological alterations in the myocardial tissues of rats were monitored. qRT-PCR, ELISA, and western blot measured the profiles of miR-27b-3p, Peroxisomal proliferating-activated receptor gamma (PPARG), inflammatory cytokines (TNF-α, IL-1β, IL-6, IL-8), and inflammatory response proteins (NF-κB-p65, MAPK-p38, JNK1/2). Besides, miR-27b-3p mimics were transfected into cardiomyocytes, and the proliferation and apoptosis of cardiomyocytes were examined through MTT and flow cytometry. As evidenced by the experimental outcomes, chrysophanol suppressed sepsis-mediated acute myocardial injury and LPS-mediated apoptosis in myocardial cells and lessened the release of pro-inflammatory cytokines and inflammatory response proteins. Moreover, chrysophanol cramped miR-27b-3p expression and heightened PPARG expression. miR-27b-3p targeted PPARG and restrained its expression. On the other hand, the PPARG agonist (RGZ) partially eliminated the apoptosis and pro-inflammatory responses of myocardial cells elicited by LPS. Therefore, this study revealed that Chrysophanol guarded against sepsis-mediated acute myocardial injury through dampening inflammation and apoptosis via the miR-27b-3p-PPARG axis, adding to the references for treating sepsis-AMI.

## Highlights

- CHR protects the heart from sepsis induced inflammatory damage;
- CHR inhibited miR-27b-3p and enhanced PPARG expression;
- miR-27b-3p promoted myocardial injury via targeting PPARG.

The article "Chrysophanol exerts a protective effect against sepsis-induced acute myocardial injury through modulating the microRNA-27b-3p/Peroxisomal proliferating-activated receptor gamma axis" was retracted in 2026. Reasons: concerns about the data; concerns about the results or conclusions.

## 1. Introduction

Sepsis, a life-threatening organ dysfunction, occurs when a patient manifests disordered responses to infection. The mortality rate of patients suffering from severe sepsis was as high as 50% worldwide in 2012 [1]. The heart is one of the important target organs for septicemic injury, which features normal or low filling pressure left ventricular dilatation, decreased ejection fraction, and reversal after 7–10 days [2]. The mortality rate of patients with post-sepsis cardiac dysfunction is four times more than that of patients with cardiomyopathy alone [3]. At present, the treatment of sepsis acute myocardial injury (S-AMI) revolves around drug thrombolysis and percutaneous coronary intervention. Notwithstanding, post-ischemic reperfusion may exacerbate the original tissue damage. Thus, there is an urgent need to develop new treatment strategies for improving the poor prognosis of S-AMI patients.

Chrysophanol (CHR) is known as a natural anthraquinone derived from the 1, 8-dihydroxyl 3-methyl derivative of the 9, 10-anthrdione ring, which mainly exists in the roots, leaves, and flowers of plants. CHR boasts a wide range of pharmacological effects like anti-tumor, anti-inflammation, anti-virus, lipid lowering, anti-diabetes, nerve protection, and liver protection [4]. CHR intervention impedes reactive oxygen species (ROS) production, abates the migration, invasion, and epithelial-mesenchymal transition of cancer cells, and bolsters the cell cycle G1 block, which is a candidate for oral cancer treatment [5]. CHR also treats neurodegenerative diseases by resisting inflammatory factor release and DNA oxidation in BV2 mouse microglia [6]. Moreover, CHR represses doxorubicin-elicited myocardial apoptosis, mitochondrial injury and augments PARylation, exerting a cardiac protective function [7]. Nevertheless, we are still in the dark about the role of CHR in S-AMI.

MicroRNAs (miRNAs), small non-coding RNAs with 22 nucleotides in length, can foster various pathophysiological processes like cell proliferation and inflammation [8], though lacking the protein-coding ability. These days, umpteen miRNAs have been identified as underlying biomarkers for sepsis [9]. Reportedly, miR-122-5p inhibition targets GIT1 to hamper inflammation and oxidative stress, hence ameliorating sepsis-triggered myocardial damage [10]. miR-21-3p can boost myocardial damage incurred by sepsis [11]. miR-27b-3p is a miRNA that emerged in recent years. In addition to exerting anti-cancer functions, miR-27b-3p is correlated with inflammation. Recent reports show that in LPS-induced microglia, miR-27b-3p overexpression uplifts the levels of pro-inflammatory cytokines (TNF-α, IL-6, IL-1β) and facilitates cell apoptosis [12]. miR-27b-3p mitigates atrial fibrosis in rats with atrial fibrillation by targeting Wnt3a to hinder the Wnt/β-catenin pathway [13]. Notwithstanding, it remains poorly understood whether miR-27b-3p takes part in S-AMI. This paper is an initial study on the function of miR-27b-3p in S-AMI.

The article "Chrysophanol exerts a protective effect against sepsis-induced acute myocardial injury through modulating the microRNA-27b-3p/Peroxisomal proliferating-activated receptor gamma axis" was retracted in 2026. Reasons: concerns about the data; concerns about the results or conclusions.

Peroxisome proliferator-activated receptor gamma (PPARγ, PPARG), a significant one in the nuclear receptor super-family, comprises an amino-terminal activation domain, a central DNA binding domain, and a carboxy-terminal ligand binding domain, which are mainly expressed in adipocytes [14]. PPARγ participates in several biological processes, such as the sustenance of lipid and glucose homeostasis, regulation of cell proliferation, intervention in inflammatory diseases, and protection of the heart. Quercetin relieves I/R-caused myocardial damage by initiating PPARG to dampen the NF-κB pathway and bolster oxidative damage and apoptosis [15]. What’s more, PPARG activated with rosiglitazone attenuates septicemic heart damage in rats [16]. In this paper, the function of the miR-27b-3p-PPARG axis in S-AMI and its exact mechanism were researched in detail.

The results of this study indicated that CHR boosted myocardial cells’ proliferation and lessened their apoptosis, whereas miR-27b-3p overexpression exacerbated myocardial cell damage mediated by LPS. Moreover, CHR concentration-dependently cramped miR-27b-3p expression and enhanced PPARG expression. Given these findings, we conjectured that CHR hampered miR-27b-3p and elevated PPARG expression to guard against myocardial damage induced by sepsis.

## 2. Materials and methods

### 2.1 The sepsis model

The Experimental Animal Center of North Sichuan Medical College (animal license: SCXK(Chuan)2018–18) was the supplier for 40 adult Sprague-Dawley rats (female, 8–10 weeks of age, 250 ~ 280 g in weight). They were reared with free access to food and water for at least one week (22–24°C, 12-hour light/dark cycle, 50–60% humidity). Specific practical steps are as follows [17]: The rats were in abrosia for 8 h prior to surgery. Then, cecal ligation and perforation (CLP) was conducted in a sterile environment to engineer a rat sepsis model. The intraperitoneal injection of 50 mg/kg sodium pentobarbital was performed for anesthesia. Following successful anesthesia, the abdomen was cut about 2–3 cm from the midline to expose the cecum, and the end of the cecum was ligated employing a sterile 3–0 silk thread. Next, the cecum was punctured with an 18-gauge needle two times. We squeezed out slight feces and put the cecum back to the abdominal cavity. The abdominal cavity was sutured layer by layer, and sterile saline (200 μL) was transfused subcutaneously to promote rat resuscitation. The rats in the sham operation group underwent the same laparotomy, but without cecal ligation and puncture. CHR (purity 98%; diluted in warm DMSO to 20 mmol/L; MCE, MedChemexpress, USA) of different doses (25, 50, 100 mg/kg) was injected into the stomachs of the rats in the CLP+CHR group from the second day subsequent to CLP. Seventy-two hours later, the rats were euthanized, and their abdominal aortic blood (5 ml) and heart tissues were harvested for subsequent experiments. We tried to minimize the sufferings of the rats to the best of our ability in line with the Guidelines for the Care and Use of Laboratory Animals. The animal procedures had received the imprimatur from the Animal Care Committee of the First Affiliated Hospital of Kunming Medical University (Approval number: KMMUH-2021-026-4).

The article "Chrysophanol exerts a protective effect against sepsis-induced acute myocardial injury through modulating the microRNA-27b-3p/Peroxisomal proliferating-activated receptor gamma axis" was retracted in 2026. Reasons: concerns about the data; concerns about the results or conclusions.

### 2.2 Hematoxylin-eosin (HE) staining

The rat heart tissues were carefully removed and immobilized in 100 mL/L formalin solution for 48 h. The tissues were dehydrated with ethanol of a conventional gradient concentration, made transparent with xylene, embedded in paraffin, and severed into slices 4 μM in thickness. Then, the slices were dewaxed with xylene, hydrated again in gradient ethanol, and dyed with hematoxylin. After being differentiated in 1% hydrochloric acid/ethanol, the sections were redyed with 1% ammonia and stained with eosin. Following staining, they were dehydrated with gradient ethanol, **cleared** with xylene, and sealed with neutral gum. At last, a microscope (200× magnification, Nikon, Tokyo, Japan) was taken for observation [18].

### 2.3 Echocardiogram measurement

On the 24^th^, 48^th^, and 72^nd^ hours following CLP, the rats were anesthetized. Echocardiography was adopted to gauge the following parameters: cardiac output (CO), ejection fraction (EF), shortened fraction (FS), left ventricular end-systolic diameter (LVESD), and left ventricular end-diastolic diameter (LVEDD). The Technos MPX ultrasound system (ESAOTE, SpAESAOTE SpA, Italy) was introduced for two-dimensional guided M-mode echocardiography, with the above-mentioned parameters recorded [19].

### 2.4 Terminal deoxynucleotidyl transferase (TdT) dUTP nick-end labeling (TUNEL) assay

The paraffin sections of the rat heart tissues were routinely dewaxed with xylene, dehydrated with gradient ethanol, and incubated along with protease K solution (20 μg/ml, diluted in 10 mmol/L Tris/HCl, pH 7.5) for 20 min at 37°C. As per the instructions of the TUNEL detection kit (HRP-DAB, ab206386, Abcam), a working solution was administered to the cells for apoptosis examination. A fluorescence microscope was taken to monitor apoptotic cells. Positive TUNEL cells were tinted with green fluorescence, and the nuclei were tinted with blue fluorescence. Five fields were chosen from each slice, and the average percentage of apoptotic cells was calculated [20].

The article "Chrysophanol exerts a protective effect against sepsis-induced acute myocardial injury through modulating the microRNA-27b-3p/Peroxisomal proliferating-activated receptor gamma axis" was retracted in 2026. Reasons: concerns about the data; concerns about the results or conclusions.

### 2.5 Myeloperoxidase (MPO) activity determination

The mouse heart tissues were homogenized and centrifuged to produce the supernatant. The MPO colorimetric activity kit (ab105136, Abcam) was adopted to examine MPO activity [21]. The activity of MPO was presented as U/g protein.

### 2.6 Immunohistochemistry (IHC) staining

As said before [22], the rat heart tissues were subjected to IHC staining. The sections were dewaxed, hydrated, and incubated along with 3% H_2_O_2_ for 10 min at room temperature to block endogenous peroxidase activity. Prior to IHC staining, the Tris/EDTA buffer solution (pH 9.0) was utilized for heat-mediated antigen repair. Then, the slices were incubated along with the rabbit anti-MPO (ab208670, Abcam, 1:1000) antibody overnight at 4°C. Later, the HRP-labeled goat anti-rabbit IgG secondary antibody (ab6721; Abcam; 1:1,000) was given to the samples for 10 minutes’ incubation at 37°C. DAB and methyl green were taken to stain the sections, respectively. An optical microscope (Nikon) was employed for observation.

### 2.7 Quantitative reverse transcription PCR (qRT-PCR)

TRIzol reagent was employed to extract miR-27b-3p and PPARG from the H9C2 cell line. The TaKaRa PrimeScript 1st Strand cDNA Synthesis Kit (TaKaRa Bio Inc, Japan) was adopted to reverse-transcribe miR-27b-3p and PPARG into cDNA. SYBR Green qPCR Master Mix (MedChemExpress, NJ, USA) and the IQ5 Multicolor qRT-PCR Detection System (Bio-Rad, USA) were utilized for real-time fluorescent quantitative PCR. The relative expression was calculated based on the 2^−ΔΔCT^ value of each gene, and all experiments were repeated 3 times. GAPDH and U6 were taken as the internal parameters of PPARG and miR-27b-3p, respectively [23]. The primer sequences are detailed in Table 1.

**Table 1.** The sequence of each molecular primer

Genes	Primer sequences (5’‐3’)	
PPARG	Forward	TTTCCTGTCAAGATCGCCCT
	Reverse	TTGCAGTGGGGATGTCTCAT
miR-27b-3p	Forward	AGGGTTCACAGTGGCTAAG
	Reverse	GAGAGGAGAGGAAGAGGGAA
GAPDH	Forward	TGTGTCCGTCGTGGATCTGA
	Reverse	TTGCTGTTGAAGTCGCAGGAG
U6	Forward	CTCGCTTCGGCAGCACA
	Reverse	AACGCTCTCACGAATTTGCGT

### 2.8 Cell treatments and transfection

American Type Culture Collection (ATCC, Rockville, MD, USA) provided the rat embryonic cardiomyocytes H9C2. The cells were placed in an RPMI1640 (Thermo Fisher Scientific, MA, USA) medium supplemented with 10% fetal bovine serum (Biowest SAS, Niayet, France) and 1% penicillin/streptomycin (Gibco, Grand Island, NY) and cultured in an incubator (37°C, 5% CO_2_). We treated the cells with LPS (Cat no: L4268, Sigma) (10, 15, 20, 25, 30 μg/mL) for 24 h and adopted the appropriate concentrations (10 μg/mL) to construct a cell damage model [24]. Lipofectamine 2000 (Thermo Fisher Scientific, Waltham, USA) was applied to transfect miR-27b-3p mimics and their corresponding negative control. CHR (purity 98%; diluted in warm DMSO to 20 mmol/L; MCE, MedChemexpress, USA) was taken to treat H9C2 cells at 20–80 μM, and the PPARG activator Rosiglitazone (RGZ, cat.no.BRL 49653, MedChemexpress, USA) was administered at 100 nM.

The article "Chrysophanol exerts a protective effect against sepsis-induced acute myocardial injury through modulating the microRNA-27b-3p/Peroxisomal proliferating-activated receptor gamma axis" was retracted in 2026. Reasons: concerns about the data; concerns about the results or conclusions.

### 2.9 Enzyme-linked immunosorbent assay (ELISA)

With a lysis buffer administered, the tissue homogenate obtained from the rat tissues underwent centrifugation at 4°C (1000 × g, 10 min). The supernatant was harvested following the centrifugation. H9C2 cells were cultured at 4°C (48 h). Then, the culture medium was collected and centrifuged (2000 r/min, 10 min). The supernatant was obtained. Finally, the ELISA kit (R&D Systems Inc., Minneapolis, USA) was exploited to confirm the profiles of pro-inflammatory cytokines (TNF-α, IL-1β, IL-6, IL-8) in the rat tissues and H9C2 cells. Additionally, the rats’ blood from the abdominal aorta was harvested. As instructed by the supplier, the concentrations of myocardial damage markers cardiac troponin I (cTnI), brain natriuretic peptide (BNP), and creatine kinase isoenzyme (CK-MB) were gauged (Beckman Coulter Life Sciences, Brea, CA, USA) [25].

### 2.10 Western blot

The rat heart tissues and H2C9 cells were treated with various factors. Then, pre-cooled RIPA lysis buffer (Beyotime Biotechnology, Shanghai, China) was adopted to extract the total protein out of the cells and tissues. The protein was centrifuged at 14,000 g (4°C) for 30 min to produce the supernatant. The Bicinchoninic Acid (BCA) protein quantification kit (Beyotime Biotechnology, Shanghai, China) was employed for protein quantification. The cell supernatant or cardiac homogenate of the comparable amount (30 µg) was separated by 12% SDS-PAGE and electrotransferred to PVDF membranes. Afterward, the membranes were sealed with 5% skimmed milk for 2 h at room temperature and cultured overnight with primary antibodies Anti-NF-kB p65 (phospho S529) antibody (ab97726, Abcam, USA, 1:1000), Anti-NF-kB p65 antibody (ab16502, Abcam, USA, 1:1000), Anti-MAPK p38 antibody (ab31828, Abcam, USA, 1:1000), Anti-MAPK p38 (phospho Y182) antibody (ab47363, Abcam, USA, 1:1000), Anti-JNK1/2 (phospho) antibody (4668, CST, USA, 1:1000), Anti-JNK1/2 antibody (9592, CST, USA, 1:1000), Anti-PPARG antibody (ab59256, Abcam, USA, 1:1000), Anti-c-Myc antibody (ab32072, Abcam, USA, 1:1000), and Anti-GAPDH antibody (ab181602, Abcam, USA, 1:1000) at 4°C. The secondary antibody Goat Anti-Rabbit IgG H&L (1:3000, ab150077, Abcam, USA) was added for hybridization (1 h, room temperature). Then, the membranes were flushed with TBST 3 times, 5 min each. GAPDH was taken as the endogenous control. Protein bands were visualized with enhanced chemical luminescence (Bio-Rad Laboratories, Inc.) and analyzed through the ImageQuant TL software (GE Healthcare, Milwaukee, WI, USA) [26].

The article "Chrysophanol exerts a protective effect against sepsis-induced acute myocardial injury through modulating the microRNA-27b-3p/Peroxisomal proliferating-activated receptor gamma axis" was retracted in 2026. Reasons: concerns about the data; concerns about the results or conclusions.

### 2.11 3-(4,5-dimethylthiazol-2-yl)-2,5-diphenyltetrazolium bromide (MTT) assay

H9C2 cells, transfected or untransfected, were inoculated into 96-well plates with a density of 2 × 10^3^/well. The cells were cultured in the presence or absence of LPS or CHR of different concentrations for 24 h. Later, 10 μL MTT solution (5 mg/mL, Sigma) was administered to each well for 2 hours’ culture at 37°C. A microplate reader (Bio-Rad, Hercules, CA, USA) was taken to gauge the absorbance value of each well at 450 nm. The experiment in each group was performed in triplicate [27].

### 2.12 Flow cytometry

FITC annexin V and Propid iumiodide were applied to examine cell apoptosis. Subsequent to trypsinization, H9C2 cells were rinsed twice with PBS and administered with 400 μL of pre-cooled PBS. Next, 10 μL of AnnexinV-FITC and 5 μL of PI were added respectively for incubation (30 min, 4°C, in the dark). A flow cytometer (Merck KGaA, Darmstadt, Germany) was taken to monitor apoptosis. The FlowLogic software (Innovai, Sydney, Australia) was introduced to analyze the percentage of apoptotic cells [28].

### 2.13 Dual luciferase activity assay

The luciferase reporter vectors (PPARG-WT and PPARG-MUT) were synthesized by Promega (Madison, WI, USA). H9C2 cells (4.5 × 10^4^) were inoculated in 48-well plates and cultured till 70% confluent. As per the instructions, lipofectamine 2000 (Thermo Fisher Scientific, Waltham, USA) was taken to co-transfect H9C2 cells with PPARG-WT or PPARG-MUT (20 nm for each), miR-27b-3p mimics or their corresponding negative control (50 nm for each). The luciferase activity was measured 48 h after transfection in keeping with the instructions of the Dual-luciferase reporter kit (Promega, Madison, WI, USA). We conducted all experiments in triplicate and repeated them three times [29].

## 2.14 5-Ethynyl-2′-deoxyuridine (EdU) assay

As described before [30], the EDU method was adopted to examine cell proliferation. Put simply, H9C2 cells, transfected or untransfected, were inoculated into 96-well plates with a density of 1x10^4^/well and treated with LPS and CHR or RGZ of different concentrations for 24 hours at 37°C with 5% CO_2_. Then, 50 μmol/L EDU solution was administered to each well for 2 hours’ incubation. PBS was utilized to flush the cells twice, which were then immobilized with 4% paraformaldehyde for 30 min. Next, 1× Apollo was given to dye the cells at room temperature and in darkness for 30 min. At last, DAPI solution (Keygen, Nanjing, China) was applied to redye the nuclei. A fluorescence microscope (Leica, Wetzlar, Germany) was operated to measure the percentage of positive EDU cells.

The article "Chrysophanol exerts a protective effect against sepsis-induced acute myocardial injury through modulating the microRNA-27b-3p/Peroxisomal proliferating-activated receptor gamma axis" was retracted in 2026. Reasons: concerns about the data; concerns about the results or conclusions.

### 2.15 Cell immunofluorescence

H9C2 cells were treated with multiple factors and immobilized in 4% paraformaldehyde for 15 min at 4°C. Next, 0.2% TritonX-100 was adopted to rinse and permeabilize the cells for 5 min at room temperature. The cells were incubated along with the anti-PPARG (ab45036, Abcam, 1:500) antibody at 4°C overnight and then with the fluorescent dye-labeled secondary antibody (1: 200, Beyotime, Shanghai, China) at room temperature for an hour. DAPI (Keygen, Nanjing, China) was taken to stain the cells in darkness for 10 min. A microscope was utilized to observe the representative images [31].

### 2.16 Statistical analysis

The GraphPad Prism 8 Software (GraphPad Software Inc., San Diego, CA, USA) was introduced for analysis. The outcomes were presented as mean ± standard deviation (x ± s). If P < 0.05, the statistics were regarded as meaningful. One-way ANOVA was implemented for comparison among multiple groups, and two independent sample t-test was conducted to compare two groups.

## 3. Results

In this study, we tried to investigate the protective role of CHR against sepsis-mediated acute myocardial injury. We found that CHR relieved LPS-mediated apoptosis and inflammation, and also mitigated CLP-induced heart damage. CHR reduced miR-27b-3p and promoted PPARG pathway activation. MiR-27b-3p, as indicated by bioinformatic analysis, is a potential upstream target of PPARG. Therefore, we supposed that CHR exerts protective effects in cardiomyocyte by regulating miR-27b-3p/PPARG axis.

### 3.1 CHR defended cardiomyocytes from LPS-induced acute myocardium injury

To confirm the impact of CHR on H9C2 cells, we treated the cells with CHR (1, 5, 25, 50, 100 μM) and discovered that CHR exerted no cytotoxicity in H9C2 cells when its concentration was below 100 μM (*P > 0.05*, Figure 1a). LPS of different concentrations (10, 15, 20, 25, 30 μg/mL) was taken to treat H9C2 cells. MTT and EdU measured cell viability and proliferation, respectively. Statistics revealed that LPS concentration-dependently hampered cell viability and proliferation (*P > 0.05*, Figure 1b-c). LPS (10 μg/mL) was employed to treat the cells for 24 h, and they were then treated with CHR (20, 40, 80 μM). Flow cytometry examined cell apoptosis, indicating that under CHR treatment, the apoptosis of H9C2 cells was remarkably lessened (in contrast with the LPS group, *P < 0.05*, Figure 1d). ELISA demonstrated that LPS remarkably up-regulated pro-inflammatory cytokines (TNF-α, IL-1β, IL-6, IL-8) (in contrast with the control group, Figure 1e-h). Following the application of CHR, those pro-inflammatory factors were dose-dependently decreased (*P < 0.05*, Figure 1e-h). Western blot exhibited that LPS enhanced NF-κB, MAPK, and JNK1/2, but in contrast with the LPS group, CHR suppressed the profiles of NF-κB, MAPK, and JNK1/2 dose-dependently (*P < 0.05*, Figure 1i). These phenomena suggested that CHR alleviated myocardial cell damage elicited by LPS.

The article "Chrysophanol exerts a protective effect against sepsis-induced acute myocardial injury through modulating the microRNA-27b-3p/Peroxisomal proliferating-activated receptor gamma axis" was retracted in 2026. Reasons: concerns about the data; concerns about the results or conclusions.

**Figure 1.** CHR defended cardiomyocytes from LPS damage Different concentrations of CHR (1, 5, 25, 50, 100 μ M) was dealt with H9c2 cells. A: cell viability was detected by MTT. H9C2 cells were treated with LPS (10–25 μg/ml) for 24 h to induce an *in-vitro* model of S-AMI. B: MTT examined cell viability; C: Edu assay detected cell viability. CHR was utilized to treat H9C2 cells at different concentrations (20 μM, 40 μM, 80 μM). D: Flow cytometry monitored cell apoptosis; E-H: ELISA measured pro-inflammatory factors’ levels in H9C2 cells; I: Western blot was taken to analyze the profiles of pro-inflammatory proteins NF-κB-p65, MAPK-p38, JNK1/2 in H9C2 cells. NS *P* > 0.05,**P < 0.01, ***P < 0.001 (vs. the control group); #*P* < 0.05, ##*P* < 0.01, ###*P* < 0.001 (vs. the LPS group). N = 3.

### 3.2 CHR ameliorated myocardial injury in sepsis rats

To investigate the protective influence of CHR on sepsis-caused myocardial damage *in vivo*, we engineered an *in-vivo* sepsis myocardial damage model with the use of CLP. During the 24 hours following CLP, CHR (25, 50, 100 mg/kg) was adopted to treat the rats. ELISA examined the profiles of myocardial injury markers (CK-MB, cTnI, BNP) in the rat serum on the 24^th^, 48^th^, and 72^nd^ hours subsequent to CLP. It turned out that in contrast with the sham group, the CLP group witnessed a distinct rise in the levels of CK-MB, cTnI, and BNP, whereas CHR gave rise to a decline in their levels (*P < 0.05*, Figure 2a). Echocardiography was employed to check cardiac output (CO), ejection fraction (EF), shortened fraction (FS), left ventricular end diastolic diameter (LVEDD) and left ventricular end-systolic diameter (LVESD) at the 24th, 48th, and 72th hour after CLP. CLP reduced CO, EF, FS, and enhanced LVIDd, . By contrast to the CLP group, CHR apparently heightened CO (*P < 0.05*, Figure 2b). The trend of EF was aligned with that of FS. Both of them hit the lowest on the 24^th^ hours following the operation, but CHR considerably elevated them (*P < 0.05*, Figure 2c-d). The values of LVIDd and LVISd were remarkably higher than those in the sham group, but in contrast with the CLP group, CHR of different concentrations brought down their levels (*P < 0.05*, Figure 2e-f). The parasternal long axis view (Figure 2g). HE staining monitored pathological alterations in the heart tissues, denoting that the rats’ myocardial structure in the sham group was normal, with clear horizontal stripes and neat cells. In the CLP group, myocardial cells were denaturated, some muscle fibers were disordered in company with interstitial edema, and inflammatory cell infiltration and hyperemia occurred. However, CHR ameliorated the CLP-triggered denaturation of the rat myocardial tissues (Figure 2h). Moreover, we conducted TUNEL and MPO assays to evaluate cell apoptosis and neutrophil infiltration. It was discovered that CLP induced obvious TUNEL-labeled apoptotic cells and MPO-labeled neutrophils (Figure 2i-j). With the administration of CHR, TUNEL-labeled apoptotic cells and MPO-labeled neutrophils were both notably lessened (by contrast to the CLP group, P < 0.05, Figure 2i-j). The above data suggested that CHR cramped myocardial injury in sepsis rats.

The article "Chrysophanol exerts a protective effect against sepsis-induced acute myocardial injury through modulating the microRNA-27b-3p/Peroxisomal proliferating-activated receptor gamma axis" was retracted in 2026. Reasons: concerns about the data; concerns about the results or conclusions.

**Figure 2.** CHR attenuated myocardial damage in sepsis rats A CLP surgery was performed on rats for constructing a rat sepsis model. CHR was administered at different doses (25, 50, 100 mg/kg). A: ELISA was used for evaluating serum myocardial injury markers (CK-MB, cTnI, BNP). B-F: cardiac output (CO), ejection fraction (EF), shortening fraction (FS), left ventricular end diastolic diameter (LVEDD) and left ventricular end-systolic diameter (LVESD) were measured by echocardiography 24, 48 and 72 hours after CLP. G: HE staining was preforming the pathological changes of myocardial tissues. H: TUNEL assay was used for evaluating cardiomyocyte apoptosis. J: MPO-staining was used for detecting neutrophil infiltration using immunohistochemistry, and the MPO activity in the heart was detected. ***P < 0.001 (vs. Sham group); NS *P* > 0.05, #*P* < 0.05, ##*P* < 0.01, ###*P* < 0.001 (vs. CLP group). N = 5.

### 3.3 CHR negatively modulated miR-27b-3p to boost PPARG expression

To ascertain the mechanism of CHR defending myocardial cells, we adopted LPS (10 μg/mL) to treat H9C2 cells for 24 h to engineer a sepsis myocardial cell injury model. qRT-PCR examined the profiles of miR-27b-3p and PPARG in H9C2 cells on the 24^th^, 48^th^, 72^nd^, and 96^th^ hours after LPS treatment. As a result, miR-27b-3p reached the highest level on the 24^th^ hour following the application of LPS, whereas PPARG was the lowest (Figure 3a-b). On the 24^th^ hour after LPS treated H9C2 cells, CHR (20, 40, 80 μM) was taken to treat the cells, with qRT-PCR implemented to gauge the profiles of miR-27b-3p and PPARG. In contrast with the LPS group, CHR concentration-dependently hampered miR-27b-3p expression and uplifted PPARG expression (*P < 0.05*, Figure 3c-d). Cell immunofluorescence checked PPARG expression. By contrast to the LPS group, CHR augmented the number of positive PPARG cells and strengthened the fluorescence intensity (Figure 3e). Prior works have corroborated that c-Myc is a downstream target of miR-27b-3p and negatively modulates miR-27b-3p expression [32]. Western blot determined the profiles of c-Myc and PPARG, indicating that LPS vigorously repressed their expressions, but in contrast with the LPS group, CHR uplifted their expressions (*P < 0.05*, figure 3f). Given these findings, we concluded that CHR boosted c-Myc to regulate the profile of the miR-27b-3p/PPARG pathway.

The article "Chrysophanol exerts a protective effect against sepsis-induced acute myocardial injury through modulating the microRNA-27b-3p/Peroxisomal proliferating-activated receptor gamma axis" was retracted in 2026. Reasons: concerns about the data; concerns about the results or conclusions.

**Figure 3.** CHR suppressed miR-27b-3p and enhanced PPARG H9c2 cells were treated with LPS (10 μg/ml) for 24 hours to construct the cell septic injury model. A-B: qRT-PCR was used to detect the expression of miR-27b-3p and PPARG in H9c2 cells 24, 48, 72 and 96 hours after LPS treatment. Different concentrations of Chr (20, 40, 80 μ M) were added into the H9c2 cells. C-D. The expression of miR-27b-3p and PPARG was detected by qRT-PCR. E: The expression of PPARG was detected by cellular immunofluorescence. Scale bar = 50 μm. F: The expressions of c-Myc and PPARG were detected by western blot. ** P < 0.01, ***P < 0.001(vs. control group); # P < 0.05, ##P < 0.01, ###P < 0.001 (vs. LPS group). N = 3.

### 3.4 miR-27b-3p targeted PPARG

Through Starbase bioinformatics (http://starbase.sysu.edu.cn/), we discovered that PPARG was an important downstream target of miR-27b-3p (Figure 4a). Moreover, dual-luciferase activity assay reflected that miR-27b-3p mimics exerted no substantial inhibitory impact on H9C2 cells transfected along with PPARG-MUT-luc vector but remarkably suppressed the luciferase level of those transfected with PPARG-WT vector (*P* < 0.05, Figure 4b). Cell immunofluorescence and western blot gauged PPARG expression. Following miR-27b-3p overexpression, the protein level of PPARG was vigorously restricted (compared with the miR-NC group, Figure 4c-d). Thus, we confirmed that miR-27b-3p targeted PPARG and cramped its expression.

**Figure 4.** miR-27b-3p targeted PPARG A: The Starbase database (http://starbase.sysu.edu.cn/) was introduced for predicting the base binding correlation between miR-27b-3p and PPARG; B: H9C2 cells were transfected along with the luciferase reporter vectors (PPARG-WT and PPARG-MUT) with miR-NC or miR-27b-3p mimics. Dual-luciferase activity assay evaluated the luciferase activity of H9C2 cells to confirm the correlation between miR-27b-3p and PPARG. C: The expression of PPARG was detected by cellular immunofluorescence. Scale bar = 50 μm. D: Western blot was conducted to evaluate the protein profile of PPARG in H9C2 cells transfected with miR-NC or miR-27b-3p mimics. NS *P* > 0.05, ***P < 0.001 (vs. the miR-NC group). N = 3.

The article "Chrysophanol exerts a protective effect against sepsis-induced acute myocardial injury through modulating the microRNA-27b-3p/Peroxisomal proliferating-activated receptor gamma axis" was retracted in 2026. Reasons: concerns about the data; concerns about the results or conclusions.

### 3.5 CHR protected myocardial cells from injury by regulating the miR-27b-3p/PPARG axis

To better understand the mechanism of CHR protecting myocardial cells, we transfected miR-NC and miR-27b-3p mimics into H9C2 cells. qRT-PCR examined miR-27b-3p expression, denoting that miR-27b-3p overexpression brought about a notable rise in the level of miR-27b-3p (*P* < 0.05, Figure 5a). We then treated H9C2 cells with CHR or the PPARG activator (RGC) to confirm the function of CHR in myocardial cell injury. PPARG was repressed after miR-27b-3p mimics transfection (by contrast to the LPS group), whereas CHR or Rosiglitazone (the PPARG activator) treatment bolstered PPARG expression (compared with the LPS+miR group) (Figure 5b). MTT examined cell viability, EdU monitored proliferation, and flow cytometry checked apoptosis. It transpired that in contrast with the LPS group, miR-27b-3p overexpression dampened cell viability and proliferation but boosted apoptosis. By contrast to the LPS+miR-27b-3p group, CHR or RGC strengthened cell viability and proliferation and lessened apoptosis (*P* < 0.05, Figure 5c-f). ELISA illustrated that the profiles of TNF-α, IL-1β, IL-6, and IL-8 were considerably higher in the LPS+miR group than in the LPS group. Their levels were down-regulated in the LPS+CHR group or the LPS+RGZ group (Figure 5g-j). Western blot unveiled that overexpression of miR-27b-3p enhanced the activation of NF-κB, MAPK, and JNK1/2 (in contrast with the LPS group, Figure 5k). In the LPS+miR+CHR and LPS+miR+RGZ groups, the activation of NF-κB, MAPK, and JNK1/2 elicited by miR-27b-3p was repressed (Figure 5k). Thus, CHR could resist inflammatory activation by suppressing miR-27b-3p.

**Figure 5.** CHR protected cardiomyocytes against LPS-mediated injury by modulating the miR-27b-3p/PPARG axis After the construction of the H9C2 cell injury model with the use of LPS (10 μg/ml), CHR (20 μM) and RGZ (100 nM) were adopted to treat the cells. A. H9C2 cells were transfected along with miR-27b-3p mimics or miR-NC, and miR-27b-3p’s level was gauged via RT-PCR. CHR was administered after miR-27b-3p mimics transfection in H9C2 cells. B: Western blot measured PPARG; C: MTT checked cell viability. D: EdU assay detected cell proliferation. E-F: Flow cytometry checked cell apoptosis, respectively; G-J: ELISA was applied to confirm the profiles of pro-inflammatory factors; K: Western blot verified the levels of pro-inflammatory proteins NF-κB MAPK, and JNK1/2 in H9C2 cells. ***P < 0.001 (vs. the miR-NC group); ***P < 0.001 (vs. the Vector group); **P < 0.01, ***P < 0.001 (vs. the NC group); #*P* < 0.05, ##*P* < 0.01 (vs. the LPS group); &&*P* < 0.01, &&&*P* < 0.001 (vs. the LPS+miR-27b-3p group). N = 3.

The article "Chrysophanol exerts a protective effect against sepsis-induced acute myocardial injury through modulating the microRNA-27b-3p/Peroxisomal proliferating-activated receptor gamma axis" was retracted in 2026. Reasons: concerns about the data; concerns about the results or conclusions.

### 3.6 CHR reduced inflammatory myocardial damage in sepsis rats via modulating the miR-27b-3p/PPARG axis

We probed into the specific protective effect of CHR on myocardium in the sepsis rats. ELISA exhibited that in contrast with the sham group, the levels of pro-inflammatory cytokines (TNF-α, IL-1β, IL-6, IL-8) in the CLP group were heightened. Their levels were lowered in the CLP+CHR group (25, 50, 100 mg/kg) vis-a-vis the CLP group, and the down-regulation degree was heightened with the increase in the dose of CHR (*P* < 0.05, Figure 6a-d). Western blot that examined inflammatory proteins in the myocardial tissues showed that the levels of pro-inflammatory proteins (p-NF-κB/NF-κB, p-MAPK/MAPK, p-JNK1/2/P-JNK1/2) were notably higher in the CLP group than in the sham group. CHR impeded the release of pro-inflammatory substances in the sepsis rats, and such inhibition was positively correlated with the dose of CHR (*P* < 0.05, Figure 6e). Furthermore, qRT-PCR and western blot were performed to evaluate c-Myc, miR-27b-3p, and PPARG levels in the heart tissues. As the data evidenced, CLP enhanced miR-27b-3p but restrained c-Myc and PPARG (compared with the Sham group, Figure 7a-b). Notwithstanding, CHR treatment repressed miR-27b-3p’s level and boosted c-Myc and PPARG expressions (versus the CLP group, Figure 7a-b). Collectively, those data unveiled that the miR-27b-3p/PPARG axis partook in the CHR-mediated protective effects on cardiomyocytes against sepsis (Figure 8).

**Figure 6.** CHR lessened inflammatory damage in sepsis rats Cecal ligation and puncture (CLP) was operated for conducting a sepsis rat model, and the rats were subcutaneously injected with CHR (25, 50, 100 mg/kg). Seventy-two hours later, the rats were sacrificed, and their hearts were collected for histopathological examination. A-D: ELISA was implemented to analyze the levels of pro-inflammatory factors (IL-8, TNF-α, IL-6, IL-1β) in the rats; E: Western blot examined the levels of pro-inflammatory proteins NF-κB, MAPK, and JNK1/2. ***P < 0.001 (vs. the Sham group); #*P* < 0.05, ##*P* < 0.01, ###*P* < 0.001 (vs. the CLP group). N = 5.

The article "Chrysophanol exerts a protective effect against sepsis-induced acute myocardial injury through modulating the microRNA-27b-3p/Peroxisomal proliferating-activated receptor gamma axis" was retracted in 2026. Reasons: concerns about the data; concerns about the results or conclusions.

**Figure 7.** CHR attenuated miR-27b-3p and boosted PPARG expression in the sepsis rat heart Cecal ligation and puncture (CLP) was performed to engineer a sepsis rat model, and the rats were subcutaneously injected with CHR (25, 50, 100 mg/kg). Seventy-two hours later, the rats were sacrificed, and their hearts were harvested for further examination. A. RT-PCR tested miR-27b-3p expression in the heart. B. Western blot examined c-Myc and PPARG in the heart. ***P < 0.001 (vs. the Sham group); #*P* < 0.05, ##*P* < 0.01, ###*P* < 0.001 (vs. the CLP group). N = 5.

**Figure 8.** The mechanism diagram of CHR CHR treatment elevated the expression level of PPARG by repressing miR-27b-3p in the myocardium, thereby lessening myocardial cell apoptosis and inflammatory factor release, enhancing cell viability, and ultimately impeding acute myocardial injury elicited by sepsis.

## 4. Discussion

The pathological process of sepsis is sophisticated. Patients’ response to the pathogen has gone far beyond the initial infection, even to the extent of severe organ dysfunction, resulting in an increase in inpatient mortality. In the context of sepsis, 40% of patients develop cardiac dysfunction [33]. Here, this research uncovered that CHR impeded myocardial cell apoptosis by modulating the miR-27b-3p/PPARG axis. CHR lessened the release of inflammatory factors and ultimately helping achieve the goal of mitigating S-AMI.

CHR, the most abundant free anthraquinone compound, is characterized by rapid absorption and strong lipophilicity. After entering the human body, it is rapidly distributed in the heart, kidney, spleen, liver, lung, brain, and other parts [34]. Many scholars regard CHR as a new inhibitor with a variety of functions. For instance, CHR mitigated OGD-mediated neuronal cell apoptosis, and proliferation inhibition [35]. The osteoblast differentiation of MC3T3-E1 cells was promoted by CHR after activating AMP-activated protein kinase (AMPK)/Small mothers against decapentaplegic (Smad1/5/9) pathway, suggesting CHR has a role in stimulating bone development [36]. Moreover, chrysophanol-loaded micelles (CLM) improve the drug delivery system for oral bioavailability improvement and exert potent anti-chronic renal failure (CRF) activity. This method provides a basis for the clinical application of CHR [37]. Presently, our data revealed that CHR cramped CLP-induced cardiomyopathy *in vivo*, boosted the activity and reduced apoptosis of LPS-injured H9C2 cells *in vitro*, suggesting that CHR is a potential effective drug in treating sepsis-mediated heart damage.

The article "Chrysophanol exerts a protective effect against sepsis-induced acute myocardial injury through modulating the microRNA-27b-3p/Peroxisomal proliferating-activated receptor gamma axis" was retracted in 2026. Reasons: concerns about the data; concerns about the results or conclusions.

The pathogenesis of sepsis acute myocardial injury (S-AMI) pertains to oxidative stress, myocardial cell apoptosis, systolic dysfunction, and long-standing inflammation. Inflammatory responses are particularly the trigger point to the aggravation of the rational damage in heart disease, which even develops into acute heart failure [38–41]. The up-regulation of TNF-α, IL-1β, and IL-6 has been confirmed to be inextricably associated with sepsis-elicited myocardial damage [42,43]. It is acknowledged that CHR restrains the profiles of pro-inflammatory genes (TNF-α, IL-6, IL-1β) in LPS-induced hepatocellular inflammation. It is expected to be utilized in the treatment of hepatitis with fewer complications and side effects [44]. Furthermore, CHR down-regulates LPS-elicited TNF-α, IL-6, and COX-2 expressions by suppressing the activation of NF-κB and Caspase-1, helping resist colitis [45]. Other scholars have demonstrated that CHR curbs the activation of NLRP3 inflammasome and guards against brain tissue injury during cerebral ischemia/reperfusion [46]. This phenomenon suggests that CHR boasts the ability to prevent organ damage triggered by inflammation. It is worth noting that CHR also has a strong cardiac protective function. CHR alleviates isoproterenepin-induced cardiac hypertrophy by repressing JAK2/STAT3 pathway activation [47]. Nrf2 activated the antioxidant, anti-inflammatory, and anti-fibrosis abilities of CHR, thereby alleviating diabetic heart injury induced by high-fat diets [48]. Other studies display that CHR efficaciously prevents myocardial injury in diabetic mice by up-regulating SIRT1, suppressing HMGB1/NF-κB pathway activation, and reducing pro-inflammatory factor release [49]. At present, CHR cramped CLP-induced release of inflammatory factors from cardiomyocytes, this helps us understand the mechanism of CHR as an effective therapeutic agent for S-AMI.

miRNAs, short regulatory RNAs, can down-regulate the protein output of their target mRNA following transcription. Over the past years, studies have demonstrated that the abnormal functions of miRNAs can contribute to severe embryo defects [50]. miRNA imbalance is very common in sepsis-induced cardiac dysfunction. For instance, miR-328 is known as a diagnostic marker in patients suffering from sepsis, and miRNA-328 expression down-regulation vigorously restrains the profiles of cTnI, CK-MB, and pro-inflammatory factors and alleviates cardiac dysfunction in patients with sepsis [51]. Furthermore, down-regulation of miR-208-5p impedes the NF-κB/HIF-1 pathway by initiating SOCS1, thereby lessening sepsis-elicited inflammatory stimulation and myocardial damage [52]. miR-29a expression is positively correlated with septicemia myocardial injury, and overexpression of lncRNA CRNDE guards against the oxidative damage and apoptosis of myocardial tissues by hindering the miR-29a/SIRT1 axis [53]. It has been reported that miR-27b-3p expression is up-regulated in endometrial stromal cells, and ginsenoside Rg3 narrows the scope of endometrial lesions and abates fibrosis by dampening miR-27b-3p so as to prevent endometriosis [54]. Interestingly, miR-27b-3p targeting at PPARG mediates the resistance of ATC to Dox, and inhibition of miR-27b-3p is conducive to overcoming the resistance of ATC to Dox [55]. However, studies on miR-27b-3p in myocardial injury post sepsis are still insufficient. Some scholars have corroborated that miR-27b-3p is a biomarker and even a therapeutic target for stroke in the context of atrial fibrillation [56]. Our research verified that miR-27b-3p expression was notably up-regulated in LPS-treated H9C2 cells, and the transfection of miR-27b-3p repressed PPARG expression. Moreover, bioinformatics analysis confirmed that miR-27b-3p targeted and negatively regulated PPARG. CHR greatly alleviated LPS-elicited myocardial cell damage by suppressing miR-27b-3p. These findings revealed that miR-27b-3p could be an underlying therapeutic target for S-AMI.

The article "Chrysophanol exerts a protective effect against sepsis-induced acute myocardial injury through modulating the microRNA-27b-3p/Peroxisomal proliferating-activated receptor gamma axis" was retracted in 2026. Reasons: concerns about the data; concerns about the results or conclusions.

In addition to adipose tissues, PPARG consists in the endothelium, vascular smooth muscle, monocytes, macrophages, and cardiomyocytes. PPARG combines with the Retinoic acid X receptor to form a heterodimer, which then binds to the ligand to incur transcriptional activation. It is noteworthy that fatty acids and dodecanoids activate PPARG in cardiometabolic regulation [14,57]. What’s more, PPARG expression up-regulation ameliorates inflammation in CLP mice, while PPARG expression inhibition augments the levels of pro-inflammatory cytokines (TNF-α, IL-6, IL-1β) in the serum [58]. Some scholars have also revealed that PPARG activation hampers VSMC proliferation, migration, and oxidative stress via up-regulation of UCP2 expression, thus preventing and treating endometrial proliferative diseases [59]. It is an interesting fact that Chrysin has been discovered to protect the cardiac function of ischemic/reperfusion rats by initiating the PPARG/Nrf2 axis [60]. Moreover, knockdown of miR-130 boosts PPARG activation and mitigates myocardial injury resulting from myocardial infarction [61]. Other studies have shown that Hesperidin elevates PPARG expression and attenuates oxidative stress and cell apoptosis, thus enhancing the myocardial functions of diabetic rats [62]. PPARG can guard against inflammation and oxidative stress, especially myocardium injury caused by sepsis. Through experiments, we uncovered that PPARG was negatively modulated by miR-27b-3p, but overexpression of PPARG, in turn, dampened miR-27b-3p so as to reduce the increased apoptosis and proliferation of LPS-induced cardiomyocytes and weaken the inflammatory injury of cardiomyocytes.

The article "Chrysophanol exerts a protective effect against sepsis-induced acute myocardial injury through modulating the microRNA-27b-3p/Peroxisomal proliferating-activated receptor gamma axis" was retracted in 2026. Reasons: concerns about the data; concerns about the results or conclusions.

## Conclusion

All in all, our research has verified that CHR modulates the miR-27b-3p/PPARG pathway, exerting a protective function against myocardial damage triggered by sepsis, which provides us with a novel way of thinking for preventing and treating septic myocardial damage. Nevertheless, experimental samples in our research were not enough, and the experimental outcomes were all based on animals. Therefore, the samples of S-AMI patients should be added in the future so as to develop new strategies for treating S-AMI.

## Data Availability

The data sets used and analyzed during the current study are available from the corresponding author on reasonable request.

## Abbreviations

BNP, brain natriuretic peptide; cTnI, cardiac troponin I; CO, cardiac output;CHR, Chrysophanol; CK-MB, creatine kinase isoenzyme; ELISA, Enzyme-linked immunosorbent assay; HE, Hematoxylin-eosin; LVEF, LV ejection fraction; LVFS, LV fractional shortening; LVEDD, left ventricular end diastolic diameter; LVESD, left ventricular end-systolic diameter; miRNAs, MicroRNAs; MPO, Myeloperoxidase; MTT, 3-(4,5-dimethylthiazol-2-yl)-2,5-diphenyltetrazolium bromide; PPARγ/PPARG, Peroxisome proliferator-activated receptor gamma; qRT-PCR, Quantitative reverse transcription PCR; ROS, reactive oxygen species; S.AMI, sepsis acute myocardial injury; TUNEL, Terminal deoxynucleotidyl transferase (TdT) dUTP Nick-End Labeling.
